The article "PDK2 promotes chondrogenic differentiation of mesenchymal stem cells by upregulation of Sox6 and activation of JNK/MAPK/ERK pathway" was retracted in 2020. Reasons: signs of a paper mill; unreliable results or conclusions; concerns about the data; concerns about the results or conclusions.

# PDK2 promotes chondrogenic differentiation of mesenchymal stem cells by upregulation of Sox6 and activation of JNK/MAPK/ERK pathway

**DOI:** 10.1590/1414-431X20165988

**Published:** 2017-02-16

**Authors:** H. Wang, X.B. Shan, Y.J. Qiao

**Affiliations:** 1 Second Department of Orthopedics, Baodi Clinical College, Tianjin Medical University, Tianjin, China; 2 Second Department of Orthopedics, The First People's Hospital of Yibin, Yibin, China; 3 First Department of Orthopedics, 4th (Xing Yuan) Hospital of Yulin, Yulin, China

**Keywords:** Pyruvate dehydrogenase kinase isoform 2, Chondrogenic differentiation, Mesenchymal stem cell, SRY-related high mobility group-box 6, c-Jun N-terminal kinase (JNK)

## Abstract

This study was undertaken to clarify the role and mechanism of pyruvate dehydrogenase kinase isoform 2 (PDK2) in chondrogenic differentiation of mesenchymal stem cells (MSCs). MSCs were isolated from femurs and tibias of Sprague-Dawley rats, weighing 300-400 g (5 females and 5 males). Overexpression and knockdown of PDK2 were transfected into MSCs and then cell viability, adhesion and migration were assessed. Additionally, the roles of aberrant PDK2 in chondrogenesis markers SRY-related high mobility group-box 6 (Sox6), type ΙΙ procollagen gene (COL2A1), cartilage oligomeric matrix protein (COMP), aggrecan (AGC1), type ΙX procollagen gene (COL9A2) and collagen type 1 alpha 1 (COL1A1) were measured by quantitative reverse-transcription polymerase chain reaction (qRT-PCR). The expressions of c-Jun N-terminal kinase (JNK), p38 mitogen-activated protein kinase (MAPK) and extracellular regulated protein kinase (ERK) were measured. Overexpressing PDK2 promoted cell viability, adhesion and inhibited cell migration in MSCs (all P<0.05). qRT-PCR assay showed a potent increase in the mRNA expressions of all chondrogenesis markers in response to overexpressing PDK2 (P<0.01 or P<0.05). PDK2 overexpression also induced a significant accumulation in mRNA and protein expressions of JNK, p38MAPK and ERK in MSCs compared to the control (P<0.01 or P<0.05). Meanwhile, silencing PDK2 exerted the opposite effects on MSCs. This study shows a preliminary positive role and potential mechanisms of PDK2 in chondrogenic differentiation of MSCs. It lays the theoretical groundwork for uncovering the functions of PDK2 and provides a promising basis for repairing cartilage lesions in osteoarthritis.

## Introduction

Osteoarthritis (OA) is a chronic joint disorder characterized by multifactorial degeneration and secondary hyperostosis of the articular cartilage, resulting from age growth, obesity, strain and injury (1 [Bibr B02]–3). Currently, OA, most prevalent at the hip and knee, has been the leading causes of disability worldwide, particularly in the elderly suffering from pain and locomotor limitation (4,5). For clinical treatment, chondrogenesis is known to be significant in skeletal development of OA, which is mainly inducted by mesenchymal stem cell (MSC) condensation and differentiation into chondrocytes (6 [Bibr B07]–8). Bone marrow MSCs exert the ability of multi-differentiation, such as chondrocytes, osteoblasts and adipocytes, and have been the common seed cells for clinical research and therapy in orthopedics field (9). As chondrogenic differentiation hardly occurs spontaneously, unveiling regulatory mechanisms regulating the differentiation from MSCs to chondrocytes in depth is an important contribution for cartilage injury repair in OA.

The article "PDK2 promotes chondrogenic differentiation of mesenchymal stem cells by upregulation of Sox6 and activation of JNK/MAPK/ERK pathway" was retracted in 2020. Reasons: signs of a paper mill; unreliable results or conclusions; concerns about the data; concerns about the results or conclusions.

Pyruvate dehydrogenase kinase (PDK) enhances phosphorylation and inactivation of the pyruvate dehydrogenase complex, which occupies a strategic role in various substrate and hormonal processes (10). PDK isoform 2 (PDK2) is one of the four PDK isoenzymes identified in mammalian tissues (11). Available evidence showed that PDK2 had considerable regulatory implications for hormonal and nutritional conditions in response to starvation, diabetes and in human muscle cells (12 [Bibr B13]–14). However, there are few reports about the effects of PDK2-meditated chondrogenic differentiation.

In the current study, to determine the role of PDK2 in directed chondrogenic differentiation from MSCs to chondrocytes, we focused on the characterization of aberrant PDK2, its effects on MSCs functions and on the potential regulatory genes and pathways.

## Material and Methods

### Cell culture

Adult male Sprague-Dawley rats (Shanghai Sipper-BK Lab Animal Co. Ltd., China), weighing 300-400 g (5 females and 5 males), were enrolled in the study. MSCs were isolated from femurs and tibias of rats according to standard procedures (15,16). All animal work followed the Ethical Guidelines and was approved by the Institutional Animal Control and Utilization Committee. MSCs were cultured in Dulbecco’s modified Eagle’s medium (DMEM; Gibco-BRL, USA) containing 10% fetal bovine serum (FBS; Gibco, USA), and incubated in a humidified atmosphere with 5% CO_2_ at 37°C.

### Lentivirus vectors construction

pBABE-puro, pBABE-puro-PDK2 (pBABE-PDK2; Addgene, USA) and lentivirus-encoded short hairpin RNA (shRNA)-PDK2, shRNA-negative control (shNC) (Open Biosystems, Inc., USA) were constructed with BLOCK-iT U6 RNAi entry vector kit (Invitrogen, USA). MSCs were transfected with lentivirus in serum-free DMEM at 37°C for 4 h. Then, 10% DMEM was added to culture MSCs for the further studies.

### Cell viability assay

After pBABEs and shRNAs transfection for 2 days, the cell viability of MSCs (10^3^ cells/well) was examined. The analysis was performed by adding 10 mg/mL 3-(4,5-dimethylthiazol-2-yl)-2, 5-diphenyltetrazolium bromide (MTT; Sigma-Aldrich, USA) to cultured medium for 4 h. Afterwards 100 μL dimethyl sulfoxide (DMSO; Lonza, USA) was employed to dissolve the blue formazan (Sigma, USA) product for 1 h. The percentage of living MSCs was recorded for 9 consecutive days at 590 nm using a Multiskan EX (Thermo Electron Corporation, USA).

The article "PDK2 promotes chondrogenic differentiation of mesenchymal stem cells by upregulation of Sox6 and activation of JNK/MAPK/ERK pathway" was retracted in 2020. Reasons: signs of a paper mill; unreliable results or conclusions; concerns about the data; concerns about the results or conclusions.

### Adhesion assay

Cell adhesion in pBABE-puro, pBABE-PDK2, shNC and shPDK2 groups was assessed with the Cell Adhesion Assay kit (Cell Biolabs, USA) according to manufacturer’s instructions. In brief, MSCs were trypsinized and added to Matrigel coated inserts (BD Bioscience, USA) in DMEM containing 2% FBS as well as 5 ng/mL transforming growth factor beta 1 (TGF-β1; Sino Biologicals, China) for 1 day. Subsequently, attached MSCs were mounted in 4% paraformaldehyde with 4,6-diamidino-2-phenylindole (DAPI; SouthernBiotech, USA) for 10 min. Inoculated MSCs were observed by absorbance at 560 nm under the DigiScan microplate reader (ASYS Hitech, Austria).

### Migration assays

The two-chamber Transwell system with an 8-μm size pore (Costar, USA) was applied to evaluate cell migration of MSCs with PDK2 overexpression or knockdown. For migration analysis, after MSCs were trypsinized (0.25% trypsin; Sigma) and suspended, they were seeded on the 24-well upper chamber with 200 mL of serum-free medium. The 600 mL of DMEM containing 10% FBS was added to the bottom chamber as chemoattractant. Following incubations in 5% CO_2_ at 37°C for 1 day, traversed MSCs on the bottom surface of the filter were fixed with 4% methanol (Sigma), stained with 0.5% crystal violet (Nanjing Sunshine Biotechnology Ltd., China), and counted under a light microscope (Amersham Pharmacia Biotech, USA).

### Quantitative reverse-transcription polymerase chain reaction (qRT-PCR)

Total RNA of MSCs with PDK2 overexpression or knockdown was prepared respectively using Trizol reagent (Invitrogen) and treated with DNase I (Promega, USA). Thereafter, 2 μg RNA was used to synthesize poly-oligo (dT) primed complementary DNA (cDNA) with the RevertAid H Minus First strand Cdna Synthesis Kit (Thermo Fischer Scientific Inc., USA). QRT-PCR reactions for PDK2, SRY-related high mobility group-box 6 (Sox6), type ΙΙ procollagen gene (COL2A1), cartilage oligomeric matrix protein (COMP), aggrecan (AGC1), type ΙX procollagen gene (COL9A2), collagen type 1 alpha 1 (COL1A1), c-Jun N-terminal kinase (JNK), p38 mitogen-activated protein kinase (MAPK) and extracellular regulated protein kinase (ERK) were performed with RiboMAX Large Scale RNA Production System T7 (Promega, Germany). The specific primer sequences of PDK2 were forward, 5′ATGGCAGTCCTCCTCTCTGA′3 and reverse 5′CACCCACCCTCTTCCTAACA′3 (17). Glyceraldehyde-3-phosphate dehydrogenase (GAPDH; Abcam, UK) was used as an internal control.

The article "PDK2 promotes chondrogenic differentiation of mesenchymal stem cells by upregulation of Sox6 and activation of JNK/MAPK/ERK pathway" was retracted in 2020. Reasons: signs of a paper mill; unreliable results or conclusions; concerns about the data; concerns about the results or conclusions.

### Western blot analysis

The protein used for western blotting was extracted from MSCs with pBABE-puro, pBABE-PDK2, shNC and shPDK2 using RIPA lysis buffer (Beyotime Institute of Biotechnology, China). After that, protein content was measured with the bicinchoninic acid Protein Assay Kit (Pierce, USA). The Bio-Rad (China) Bis-Tris Gel system was established, in which primary antibodies PDK2 (ab68164), JNK (ab124956), p38 (ab31828), ERK (ab54230) and the internal control GAPDH were obtained from Abcam. The indicated primary antibodies were resolved by 5% blocking buffer (1:1000) and were cultured at 4°C overnight. The blots were revealed using secondary antibodies with horseradish peroxidase (1:2000) at 37°C for 1 h. Thereafter, reaction products and antibodies were transferred onto the polyvinylidene fluoride (PVDF; Millipore Co., USA) membrane by the semi-dry transfer method. Signals were visualized from the stained gel with gel documentation system (Gel Doc 2000; Bio-Rad).

### Statistical analysis

Experiments were carried out three times. Data are reported as means±SD. Multiple comparisons were performed by one-way ANOVA with SPSS 19.0 software (USA). Differences were considered to be statistically significant at P<0.05.

## Results

### Transfection efficiency of PDK2 overexpression and knockdown in MSCs

The pBABE-puro and pBABE-PDK2 were transfected to construct PDK2 overexpression and shRNA-PDK2, shNC were transfected to construct PDK2 knockdown with lentivirus in MSCs, respectively. The qRT-PCR was used to validate the overexpression and knockdown efficiency at PDK2 mRNA and protein levels (Figure 1). The results showed that after transfection with the pBABE-PDK2, the mRNA and protein expression of PDK2 had a remarkable increase compared to the control (Figure 1A and C, P *<*0.01). Concurrently, shRNA-PDK2 significantly reduced the mRNA and protein expression of PDK2 compared to shNC (Figure 1B and C, P *<*0.01). Thus, overexpression and knockdown of PDK2 were effective and these transferred MSCs could be used in further studies.

**Figure 1:** *A*, mRNA expression of PDK2 in MSCs by pBABE-PDK2; *B*, mRNA expression of PDK2 in MSCs by PDK2 knockdown with shPDK2; *C*, Protein expression of PDK2 in MSCs by PDK2 overexpression and knockdown. PDK2: pyruvate dehydrogenase kinase isoform 2; sh: short hairpin; NC: negative control; GAPDH: glyceraldehyde-3-phosphate dehydrogenase; MSC: mesenchymal stem cell. **P<0.01 (ANOVA).

The article "PDK2 promotes chondrogenic differentiation of mesenchymal stem cells by upregulation of Sox6 and activation of JNK/MAPK/ERK pathway" was retracted in 2020. Reasons: signs of a paper mill; unreliable results or conclusions; concerns about the data; concerns about the results or conclusions.

### PDK2 promoted cell viability, adhesion and inhibited cell migration in MSCs

Functionally, to investigate the role of PDK2 in MSCs, cell viability, adhesion and migration were assessed. We found that overexpressing PDK2 enhanced cell viability and caused a striking decrease on day 9 (P<0.05, Figure 2A), while cell viability was significantly reduced by shPDK2 compared to shNC at 9 days (P<0.05).

**Figure 2:** Effects of aberrant PDK2 on cell viability (*A*), cell adhesion (*B*) and cell migration (*C*) in MSCs. PDK2: pyruvate dehydrogenase kinase isoform 2; sh: short hairpin; NC: negative control; MSC: mesenchymal stem cell. Data are reported as means±SD. *P*<*0.05 (ANOVA).

Strong accumulation of cell adhesion was detected in response to overexpressing PDK2 compared to the control, whereas silencing PDK2 remarkably lessened the percentage of MSC adhesion (both P<0.05, Figure 2B).

The number of migratory MSCs was significantly downregulated by overexpressing PDK2 and was upregulated by shPDK2 compared with the control (both P<0.05). Accordingly, it was concluded that PDK2 promoted cell viability, adhesion and inhibited cell migration in MSCs (Figure 2C).

### PDK2 promoted chondrogenic differentiation in MSCs

Next, the mRNA expressions of chondrogenic differentiation markers were determined via qRT-PCR after MSCs were transfected with pBABE-PDK2, shRNA-PDK2 and their controls, to explore whether PDK2 exerted an effect on chondrogenic differentiation in MSCs. qRT-PCR assay of MSCs showed a potent increase in the mRNA expression levels of chondrogenesis markers including Sox6, COL2A1, COMP, AGC1, COL9A2 and COL1A1 in response to overexpressing PDK2 (P<0.01 or P<0.05, Figure 3). Besides, the observable arrest in the mRNA expressions of all markers was witnessed by silencing PDK2 (all P<0.05). The above findings revealed that PDK2 promoted early chondrogenic differentiation of MSCs.

**Figure 3:** Effects of aberrant PDK2 on mRNA expressions of chondrogenesis markers in mesenchymal stem cell. PDK2: pyruvate dehydrogenase kinase isoform 2; sh: short hairpin; NC: negative control; Sox6: SRY-related high mobility group-box 6; COL2A1: type ΙΙ procollagen gene; COMP: cartilage oligomeric matrix protein; AGC1: aggrecan; COL9A2: type ΙX procollagen gene; COL1A1: collagen type 1 alpha 1; GAPDH: glyceraldehyde-3-phosphate dehydrogenase. Data are reported as means±SD. *P<0.05; **P*<*0.01 compared with pBABE or shNC group (ANOVA).

### PDK2 upregulated JNK/MAPK/ERK pathway to promote chondrogenic differentiation of MSCs

To further understand the mechanism of PDK2 in chondrogenic differentiation of MSCs, we evaluated the impact of PDK2 on expression of key proteins in JNK/MAPK/ERK signaling pathway. Figure 4A shows that overexpressing PDK2 induced a significant accumulation in mRNA expressions of JNK, p38MAPK and ERK in MSCs compared with the control (P<0.01 or P<0.05). mRNA expressions of these markers were significantly lower with the addition of shPDK2 than with shNC (all P<0.05). Similar outcomes were observed in western blot results (Figure 4B). The protein expression of JNK, p38MAPK and ERK in MSCs was upregulated by overexpressing PDK2 and was downregulated by silencing PDK2. Collectively, it revealed that PDK2 promoted chondrogenic differentiation of MSCs by activating JNK/MAPK/ERK signaling pathway.

The article "PDK2 promotes chondrogenic differentiation of mesenchymal stem cells by upregulation of Sox6 and activation of JNK/MAPK/ERK pathway" was retracted in 2020. Reasons: signs of a paper mill; unreliable results or conclusions; concerns about the data; concerns about the results or conclusions.

**Figure 4:** PDK2 upregulation of JNK/MAPK/ERK signaling pathway in mesenchymal stem cell. PDK2: pyruvate dehydrogenase kinase isoform 2; sh: short hairpin; NC: negative control; JNK: c-Jun N-terminal kinase; ERK: extracellular regulated protein kinase; GAPDH: glyceraldehyde-3-phosphate dehydrogenase. *P<0.05; **P<0.01 compared with pBABE or shNC group (ANOVA).

## Discussion

The effects of PDK2 on chondrogenic differentiation are not yet well understood. However, this study was a preliminary investigation on whether aberrant PDK2 modulated chondrogenic differentiation of MSCs, and if so, what the molecular mechanism might be. The present study showed that PDK2 overexpression promoted MSC viability and adhesion, inhibited cell migration and promoted chondrogenic differentiation of MSCs by activating the JNK/MAPK/ERK signaling pathway. Meanwhile the PDK2 knockdown exerted the opposite effects. Hence, our study proposed that PDK2 possesses a landmark effect on chondrogenic differentiation of MSCs laying the groundwork for repairing cartilage injury in OA with MSCs.

MSCs are a population of cells with the potent ability to differentiate into osteogenic, chondrogenic or adipogenic lineages (18). Thereby, this property qualifies MSCs as breakthrough in the study of therapeutic mechanisms for lesions in mesenchymal tissues in OA patients (19). Contractor et al. (20) linked PDK2 to key tumor factors such as p53 and reinforced that PDK2 played a role in breast cancer. In addition, there is a report corroborating that the inhibition of PDK2 by small interfering RNA (siRNA) induced apoptosis, decreased proliferation, and suppressed tumor growth of non-small-cell lung cancer (21). Thus, it is concluded that ectopic expression of PDK2 could modulate many functions of MSCs, such as cell viability, adhesion and migration, which might correlate with directed differentiation to chondrocytes.

Recently, the chondrogenic differentiation of MSCs has been reported to be regulated by several transcription and growth factors, mainly by the Sox family. Sox6 is known as a primary marker of chondrogenesis and osteogenesis of human bone marrow MSCs by driving the mesenchymal condensation and differentiation (22 [Bibr B23] [Bibr B24]–25). In this study, our results showed that mRNA levels of Sox6 were upregulated by overexpressing PDK2 and downregulated by silencing PDK2 in rat MSCs.

The article "PDK2 promotes chondrogenic differentiation of mesenchymal stem cells by upregulation of Sox6 and activation of JNK/MAPK/ERK pathway" was retracted in 2020. Reasons: signs of a paper mill; unreliable results or conclusions; concerns about the data; concerns about the results or conclusions.

To recapitulate the mechanism of PDK2-mediated chondrogenic differentiation in MSCs, we evaluated the impact of aberrant PDK2 on key proteins of MAPK pathways. We observed that PDK2 promoted phosphorylation of MAPKs in MSCs. It is well known that MAPKs, comprising JNK, p38, ERK and ERK5 pathways, are involved in various biological developments and processes (26). Moreover, previous evidence has pointed that JNK mediated the induction of autophagic cell death in numerous types of tumors (27 [Bibr B28]–29) and MAPKs might activate the mitochondrial pathway (30). In this study, the qRT-PCR and western blotting assay revealed that PDK2 could activate the JNK/MAPK/ERK pathway, which explained the PDK2 promotion of MSC viability and cell migration inhibition. Thereby, our data indicated that the PDK2-mediated activation of chondrogenic differentiation was via activation of JNK/MAPK/ERK signaling pathways.

Overexpression of endogenous PDK2 in MSCs by transfection of pBABE-PDK2 resulted in enhancement of chondrogenic differentiation as shown by a significant increase in chondrogenesis markers at mRNA level. The results of qRT-PCR showed that modulation of PDK2 potently affected the mRNA expression of key genes related to chondrocyte. Taken together, our data indicates that PDK2 acted as a key positive regulator of early chondrogenic differentiation of MSCs, and it might be a novel therapeutic biomarker for OA.

Growing evidence suggests that overexpressing PDK2, in line with higher pyruvate dehydrogenase alpha subunit (PDHα) phosphorylation status, is related to increased lactate production displayed by rat brain astrocytes (31) and breast cancer MCF7 cells (20). Thereby, it is speculated that aberrant PDK2 may regulate lactate accumulation and cytosolic pH acidification in MSCs. Since the PDK2-mediated chondrogenic differentiation was evidenced by our work, future research is warranted to determine entire effects of PDK2 on MSCs, especially on lactate synthesis, secretion and extracellular pH regulation, as well as its underlying mechanism.

In summary, this study shows a preliminary detection of a positive role and potential mechanisms of PDK2 in chondrogenic differentiation of MSCs. It lays the theoretical groundwork for uncovering the functions of PDK2 in depth and provides a promising basis for repairing cartilage injury in OA patients.

The article "PDK2 promotes chondrogenic differentiation of mesenchymal stem cells by upregulation of Sox6 and activation of JNK/MAPK/ERK pathway" was retracted in 2020. Reasons: signs of a paper mill; unreliable results or conclusions; concerns about the data; concerns about the results or conclusions.

## References

[1] Felson DT, Lawrence RC, Dieppe PA, Hirsch R, Helmick CG, Jordan JM (2000). Osteoarthritis: new insights. Part 1: The disease and its risk factors. Ann Int Med.

[B02] Johnson VL, Roe JP, Salmon LJ, Pinczewski LA, Hunter DJ (2016). Does age influence the risk of incident knee osteoarthritis after a traumatic anterior cruciate ligament injury?. Am J Sports Med.

[3] Maerz T, Newton MD, Kurdziel MD, Altman P, Anderson K, Matthew HW (2016). Articular cartilage degeneration following anterior cruciate ligament injury: a comparison of surgical transection and noninvasive rupture as preclinical models of post-traumatic osteoarthritis. Osteoarthritis and Cartilage.

[4] Woolf AD, Pfleger B (2003). Burden of major musculoskeletal conditions. Bull World Health Organ.

[5] Lin CW, Taylor D, Bierma-Zeinstra SM, Maher CG (2010). Exercise for osteoarthritis of the knee. Phys Ther.

[6] Lee S, Yoon DS, Paik S, Lee KM, Jang Y, Lee JW (2014). microRNA-495 inhibits chondrogenic differentiation in human mesenchymal stem cells by targeting Sox9. Stem Cells Develop.

[B07] Tang C, Jin C, Xu Y, Wei B, Wang L (2016). Chondrogenic differentiation could be induced by autologous bone marrow mesenchymal stem cell-derived extracellular matrix scaffolds without exogenous growth factor. Tissue Engin Part A.

[8] Boucher H, Vanneaux V, Domet T, Parouchev A, Larghero J (2016). Circadian clock genes modulate human bone marrow mesenchymal stem cell differentiation, migration and cell cycle. PloS One.

[9] Yang B, Guo H, Zhang Y, Chen L, Ying D, Dong S (2011). MicroRNA-145 regulates chondrogenic differentiation of mesenchymal stem cells by targeting Sox9. PloS One.

[10] Sugden MC, Holness MJ (1994). Interactive regulation of the pyruvate dehydrogenase complex and the carnitine palmitoyltransferase system. FASEB J.

[11] Bowker-Kinley MM, Davis WI, Wu P, Harris RA, Popov KM (1998). Evidence for existence of tissue-specific regulation of the mammalian pyruvate dehydrogenase complex. Biochem J.

[12] Holness MJ, Bulmer K, Smith ND, Sugden MC (2003). Investigation of potential mechanisms regulating protein expression of hepatic pyruvate dehydrogenase kinase isoforms 2 and 4 by fatty acids and thyroid hormone. Biochem J.

[B13] Huang B, Wu P, Bowker-Kinley MM, Harris RA (2002). Regulation of pyruvate dehydrogenase kinase expression by peroxisome proliferator-activated receptor-alpha ligands, glucocorticoids, and insulin. Diabetes.

[14] Abbot EL, McCormack JG, Reynet C, Hassall DG, Buchan KW, Yeaman SJ (2005). Diverging regulation of pyruvate dehydrogenase kinase isoform gene expression in cultured human muscle cells. FEBS J.

The article "PDK2 promotes chondrogenic differentiation of mesenchymal stem cells by upregulation of Sox6 and activation of JNK/MAPK/ERK pathway" was retracted in 2020. Reasons: signs of a paper mill; unreliable results or conclusions; concerns about the data; concerns about the results or conclusions.

[15] Javazon EH, Colter DC, Schwarz EJ, Prockop DJ (2001). Rat marrow stromal cells are more sensitive to plating density and expand more rapidly from single-cell-derived colonies than human marrow stromal cells. Stem Cells.

[16] Mangi AA, Noiseux N, Kong D, He H, Rezvani M, Ingwall JS (2003). Mesenchymal stem cells modified with Akt prevent remodeling and restore performance of infarcted hearts. Nature Medicine.

[17] Roh JL, Park JY, Kim EH, Jang HJ, Kwon M (2016). Activation of mitochondrial oxidation by PDK2 inhibition reverses cisplatin resistance in head and neck cancer. Cancer Letters.

[18] Pittenger MF, Mackay AM, Beck SC, Jaiswal RK, Douglas R, Mosca JD (1999). Multilineage potential of adult human mesenchymal stem cells. Science.

[19] Barry F, Boynton RE, Liu B, Murphy JM (2001). Chondrogenic differentiation of mesenchymal stem cells from bone marrow: differentiation-dependent gene expression of matrix components. Exper Cell Res.

[20] Contractor T, Harris CR (2012). p53 negatively regulates transcription of the pyruvate dehydrogenase kinase Pdk2. Cancer Res.

[21] Bonnet S, Archer SL, Allalunis-Turner J, Haromy A, Beaulieu C, Thompson R (2007). A mitochondria-K+ channel axis is suppressed in cancer and its normalization promotes apoptosis and inhibits cancer growth. Cancer Cell.

[22] Dzobo K, Turnley T, Wishart A, Rowe A, Kallmeyer K, van Vollenstee FA (2016). Fibroblast-derived extracellular matrix induces chondrogenic differentiation in human adipose-derived mesenchymal stromal/stem cells *in vitro*. Int J Mol Sci.

[B23] Yang KG, Saris DB, Geuze RE, Helm YJ, Rijen MH, Verbout AJ (2006). Impact of expansion and redifferentiation conditions on chondrogenic capacity of cultured chondrocytes. Tissue Engin.

[B24] Leung VY, Gao B, Leung KK, Melhado IG, Wynn SL, Au TY (2011). SOX9 governs differentiation stage-specific gene expression in growth plate chondrocytes via direct concomitant transactivation and repression. PLoS Genetics.

[25] Giuliani N, Lisignoli G, Magnani M, Racano C, Bolzoni M, Dalla Palma B (2013). New insights into osteogenic and chondrogenic differentiation of human bone marrow mesenchymal stem cells and their potential clinical applications for bone regeneration in pediatric orthopaedics. Stem Cells Int.

[26] Wang J, Qin Y, Mi X (2016). The protective effects of bone marrow-derived mesenchymal stem cell (BMSC) on LPS-induced acute lung injury via TLR3-mediated IFNs, MAPK and NF-kappaB signaling pathways. Biomed Pharmacother.

[27] Park KJ, Lee SH, Lee CH, Jang JY, Chung J, Kwon MH (2009). Upregulation of Beclin-1 expression and phosphorylation of Bcl-2 and p53 are involved in the JNK-mediated autophagic cell death. Biochem Biophys Res Commun.

The article "PDK2 promotes chondrogenic differentiation of mesenchymal stem cells by upregulation of Sox6 and activation of JNK/MAPK/ERK pathway" was retracted in 2020. Reasons: signs of a paper mill; unreliable results or conclusions; concerns about the data; concerns about the results or conclusions.

[B28] Shimizu S, Konishi A, Nishida Y, Mizuta T, Nishina H, Yamamoto A (2010). Involvement of JNK in the regulation of autophagic cell death. Oncogene.

[29] Zhang C, Jia X, Wang K, Bao J, Li P, Chen M (2016). Polyphyllin VII induces an autophagic cell death by activation of the JNK pathway and Inhibition of PI3K/AKT/mTOR pathway in HepG2 cells. PloS One.

[30] Hong HY, Kim BC (2007). Mixed lineage kinase 3 connects reactive oxygen species to c-Jun NH2-terminal kinase-induced mitochondrial apoptosis in genipin-treated PC3 human prostate cancer cells. Biochem Biophys Res Commun.

[31] Halim ND, McFate T, Mohyeldin A, Okagaki P, Korotchkina LG, Patel MS (2010). Phosphorylation status of pyruvate dehydrogenase distinguishes metabolic phenotypes of cultured rat brain astrocytes and neurons. Glia.

